# Identification of SMIM1 and SEZ6L2 as Potential Biomarkers for Genes Associated with Intervertebral Disc Degeneration in Pyroptosis

**DOI:** 10.1155/2022/9515571

**Published:** 2022-05-07

**Authors:** Nan Wang, Xiyu Liu, Xiaoyang Fang, Shuang Chen, Zhipeng Xi, Xiaoyu Zhang, Congyang Xue, Xin Liu, Lin Xie

**Affiliations:** Department of Spine Surgery, Affiliated Hospital of Integrated Traditional Chinese and Western Medicine, Nanjing University of Chinese Medicine, Nanjing, Jiangsu Province 210028, China

## Abstract

**Background:**

Inflammatory reactions and pyroptosis play an important role in the pathology of intervertebral disc degeneration (IDD). The aim of the present study was to investigate pyroptosis in the nucleus pulposus cells (NPCs) of inflammatory induced IDD by bioinformatic methods and to search for possible diagnostic biomarkers.

**Methods:**

Gene expression profiles related to IDD were downloaded from the GEO database to identify differentially expressed genes (DEGs) between inflammation-induced IDD and non-inflammatory intervention samples. Pyroptosis genes were then searched for, and their expression in IDD was analyzed. Weighted gene co-expression network analysis (WGCNA) was then used to search for modules of IDD genes associated with pyroptosis and intersected with DEGs to discover candidate genes that would be diagnostically valuable. A LASSO model was developed to screen for genes that met the requirements, and ROC curves were created to clarify the diagnostic value of the genetic markers. Ultimately, the screened genes were further validated, and their diagnostic value assessed by selecting gene sets from the GEO database. RT-PCR was used to assess the mRNA expression of diagnostic markers in the nucleus pulposus (NP). Pan-cancer analysis was applied to demonstrate the expression and prognostic value of the screened genes in various tumors.

**Results:**

A total of 733 DEGs were identified in GSE41883 and GSE27494, which were mainly enriched in transmembrane receptor protein serine/threonine, kinase signaling pathway, response to lipopolysaccharide, and other biological processes, and they were mainly related to TGF beta signaling pathway, toll-like receptor signaling pathway, and TNF signaling pathway. A total of 81 genes related to pyroptosis were identified in the literature, and eight genes related to IDD were identified in the Veen diagram, namely, IL1A, IL1B, NOD2, GBP1, IL6, AK1, EEF2K, and PYCARD. Eleven candidate genes were obtained after locating the intersection of pyroptosis-related module genes and DEGs according to WGCNA analysis. A total of six valid genes were obtained after constructing a machine learning model, and five key genes were finally identified after correlation analysis. GSE23132 and GSE56081 validated the candidate genes, and the final IDD-related diagnostic markers were obtained as SMIM1 and SEZ6L2. RT-PCR results indicated that the mRNA expression of both was significantly elevated in IDD. The pan-cancer analysis demonstrated that SMIM1 and SEZ6L2 have important roles in the expression and prognosis of various tumors.

**Conclusion:**

In conclusion, this research identifies SMIM1 and SEZ6L2 as important biomarkers of IDD associated with pyroptosis, which will help to unravel the development and pathogenesis of IDD and determine potential therapeutic targets.

## 1. Introduction

Intervertebral disc degeneration (IDD) is a chronic degenerative disease that is an important cause of chronic back and leg pain and even disability [1, 2]. Studies have shown that approximately 40% of people under the age of 30 and over 90% of people over 55 years old worldwide have varying degrees of IDD [3]. With an aging population, IDD is becoming a major threat to social development and places a huge physical and psychological burden on patients [4, 5]. IDD is dangerous in clinical practice and can cause a range of intractable conditions such as lumbar disc herniation (LDH), discogenic pain (DP), lumbar spinal stenosis (LSS), cervical spondylosis (CS), and many others [6]. The complex pathogenesis of IDD is still not entirely known, despite modern medicine having studied it in many ways.

It has been demonstrated that the inflammatory response is an important factor in IDD [6–9]. With worsening IDD, the expression of proinflammatory factors in the nucleus pulposus (NP) increases significantly, with interleukin (IL)-1*β* and tumor necrosis factor-alpha (TNF-*α*) being the most representative [10]. Pyroptosis has been a comparatively popular mechanism in recent years. It is a programmed cell death, also known as inflammatory necrosis, closely related to inflammation, immunity, and apoptosis [11]. Various studies have shown that pyroptosis plays a crucial role in IDD [12, 13]. When NP cells (NPCs) undergo pyroptosis, the main manifestations are raised inflammatory factors, NLRP3, caspase-1, and other genes [14]. It is evident that pyroptosis plays an important role in the pathology of IDD, but the important genes and diagnostic markers associated with it are still unknown.

With the constant maturation and development of information technology and gene sequence technology, important biomarkers for some common clinical diseases have been steadily screened out and can be used as important targets for subsequent diagnosis or treatment [15]. Accordingly, this study utilizes bioinformatics techniques to retrieve differentially expressed genes (DEGs) associated with IDD from the Gene Expression Omnibus (GEO) database and then analyzes the association between them. Different analysis methods and machine learning algorithms were used to screen out important genes for IDD diagnosis. Lastly, validation with external datasets and RT-PCR to discover optimal diagnostic biomarkers provides some theoretical basis for clinical diagnosis and even therapy of LDD.

## 2. Materials and Methods

### 2.1. Data Source

The datasets for this study were all sourced from the GEO database (https://www.ncbi.nlm. http://nih.gov/geo/). We downloaded the gene expression profiles in GSE41883, GSE27494, GSE23130, GSE124272, and GSE56081. GSE41883, GSE27494, and GSE124272 were used as the training set and GSE23130 and GSE56081 as the validation set. The specific dataset information is displayed in Table 1.

### 2.2. DEGs Identification and Functional Enrichment Analysis

The R software limma package investigated differential gene expression between the two groups of samples in GSE41883 and GSE27494. “Adjusted *P* < 0.05 and log2 (FC) > 2 or log2 (FC) < −2”was defined as the threshold gene differential expression screening condition. The PCA plot was created with the R package ggord, and the heat map was presented with the R package pheatmap. To further confirm the potential function of the differential genes, GO and KEGG functional enrichment analysis was performed by the ClusterProfiler program package.

### 2.3. Pyroptosis-Related Genes and Venn Diagramming

This article included 81 genes related to pyroptosis based on previous studies [16–18]. We searched for genes associated with pyroptosis in DEGs by mapping Venn diagrams (http://bioinformatics.psb.ugent.be/webtools/Venn/).

### 2.4. WGCNA Analysis

WGCNA analysis was performed on the selected dataset using the WGCNA package in the R software. First, outliers were filtered to make the model more stable, an appropriate soft threshold *β* was selected, and the topological overlap matrix (TOM) was further constructed to generate a hierarchical clustering tree of genes using hierarchical clustering. The gene significance (GS) and module membership (MM) were calculated to measure the significance of genes and clinical information and to analyze the significant associations between modules and models.

### 2.5. Identification of Biomarkers in IDD

The modular genes obtained from WGCNA analysis were intersected with differential genes to obtain core genes associated with pyroptosis. Significant genes were then selected using the Least Absolute Shrinkage and Selection Operator (LASSO) algorithm of the glmnet package in R software. The diagnostic value of the obtained genes was clarified by plotting ROC curves. The ultimately obtained genes are of great value in the diagnosis of IDD.

### 2.6. Validation of Key Biomarkers

To clarify the expression of diagnostic markers, the specific expression of the obtained pivotal genes was validated by the independent datasets GSE23130 and GSE56081.

### 2.7. Real-Time Quantitative Polymerase Chain Reaction (RT-PCR)

The NP tissue was obtained from patients who underwent percutaneous endoscope lumbar discectomy (PELD) at the Jiangsu Provincial Hospital of Integrated Chinese and Western Medicine. All patients signed an informed consent form, and the research was approved by the Ethics Committee of the Affiliated Hospital of Integrated Traditional Chinese and Western Medicine, Nanjing University of Chinese Medicine (Ethical Lot Number: 2020LWKY023). A total of 25 patients, fourteen with mild degeneration (MD) and others with severe degeneration (SD), were included for relevant molecular biological studies. To further validate SMIM1 and SEZ6L2 mRNA levels, we executed in vitro experiments. Rat NPCs were purchased from *Procell*, and we constructed a degeneration model by IL-1*β* (10 ng/ml). NP tissue and cellular RNA were extracted utilizing the Trizol method and reverse translated into cDNA using ProtoScript II First Strand cDNA Synthesis Kit. RT- PCR was then executed on a Quanstudio DX fluorescent quantitative PCR instrument system utilizing Luna Universal qPCR Master Mix (see Table S1 for the specific primer sequence).

### 2.8. Pan-Cancer Analysis of SMIM1 and SEZ6L2

We downloaded the pan-cancer dataset from TCGA TARGET GTEx (PANCAN, *N* = 19131, *G* = 60499) in UCSC (https://xenabrowser.net/) database and extracted the expression data of SMIM1 and SEZ6L2 genes. Samples were retrieved from solid tissue normal, primary solid tumor, primary tumor, normal tissue, primary blood-derived cancer-bone marrow, and primary blood-derived cancer. Finally, we executed a log2(x + 0.001) transformation of the expression values. Differences in expression between normal and tumor samples were calculated by R software and subsequently analyzed for the significance of differences using a nonparametric test.

### 2.9. Prognosis and Survival Analysis

TCGA prognostic dataset the cited from a high-quality research article published in Cell in 2018 [19]. TARGET follow-up data were obtained from the UCSC Cancer Browser (https://xenabrowser.net/datapages/). The Cox proportional hazards regression model was constructed by the coxph function of the survival package in R software to evaluate the prognostic relationship between SMIM1 and SEZ6L2 with pan-cancer [20]. The optimal cutoff values for SMIM1 and SEZ6L2 were calculated using the maxstat package, setting the minimum grouping sample size greater than 25% and the maximum sample size grouping less than 75%, splitting the patients into two groups based on the cutoff values.

### 2.10. Statistical Analysis

All data were statistically analyzed using R and Graph Pad Prism. Measures were expressed as a nonparametric test to compare differences between the two groups, with *P* < 0.05 indicating a significant difference.

## 3. Results

### 3.1. Identification of DEGs

GSE41883 and GSE27494 were combined, the microarray data were homogenized (Figure 1(a)), and PCA analysis was performed to clarify sample correlation (Figures 1(b) and 1(c)). A total of 733 DEGs were identified after a differential analysis of the microarray data, including 416 upregulated genes and 317 downregulated genes, the results of which were shown by the volcano plot (Figure 1(d)). The expression of the differential genes was displayed in a heat map (Figure 1(e)). GO and KEGG enrichment analyses were performed on up- and downregulated DEGs, respectively, to clarify their biological functions (Figure 2).

### 3.2. Identification of Pyroptosis in IDD

Pyroptosis has been demonstrated to play an important role in IDD. Consequently, we searched for 81 pyroptosis (Table S2) related genes and took intersections between DEGs. The five upregulated genes, namely, IL1A, IL1B, NOD2, GBP1, and IL6 (Figure 3(a)), and three downregulated genes, namely, AK1, EEF2K, and PYCARD (Figure 3(b)), were obtained.

### 3.3. Identification of Pyroptosis-Related Gene Modules

We performed WGCNA analysis on the GSE124272 dataset to further explore the genes associated with the pyroptosis module. Using the WGCNA package of the R software, we constructed the model (Figure 4(a)), and by using the pick Soft Threshold function, we found the best soft threshold for this model to be 30, where R2 was 0.87 (Figure 4(c)) and mean connectivity was 14.48 (Figure 4(d)). After merging similar modules, this model forms eight different modules (Figure 4(b)). We then correlated the coexpression modules and found that the dark grey and ivory modules were more in line with our requirements (see Figure 4(e) for a heat map of module and phenotype correlations and Figure 5 for a scatter plot of GS and MM correlations).

### 3.4. Acquisition of key Biomarkers for IDD

The DEGs of GSE124272 were obtained by limma package, and 188 differential genes were obtained (Figure S1). It was intersected with the gene modules obtained by WGCNA to obtain a total of 11 related genes, namely, SMIM1, FBLN2, ZFP2, B4GALT5, HCRT SLC6A17, MUSK, SLC26A8, CRHR2, SEZ6L2, and KCNJ15 (Figure 6(a)). The 11 obtained genes were subjected to correlation analysis (Figure 6(c)), and B4GALT5 was not highly correlated with other genes and was thus excluded. The remaining 10 relevant genes were then input into LASSO utilizing a machine learning approach to attain high diagnostic value gene markers. After LASSO coefficient profiles (Figure 6(b)) and validation (Figure 6(d)), five candidate markers were obtained, namely, “SMIM1,” “FBLN2,” “ZFP2,” “SLC6A17,” and “SEZ6L2.” The ROC curves were then plotted to demonstrate the validity of the candidate genes (Figure 6(e)), and the areas under the curves were found to be 0.828, 0875, 0.891, 0.797, and 0.797, respectively, implying that it was highly accurate.

### 3.5. Verification of the Key Biomarkers for IDD

In order to verify the correlation between the candidate genes and improve the diagnostic value, we conducted correlation analysis on the selected genes (Figure 7(a)) and found that they were significantly associated with each other. Subsequently, to validate the validity of the candidate genes, we involved the external datasets GSE23130 and GSE56081 to identify differential expression between the two groups. We found that GSE23130, SMIM1, SLC6A17, and SEZ6L2 were all differentially altered in the SD compared to the MD group, and the differences were statistically significant (Figure 7(b)). In addition, SMIM1, ZFP2, and SEZ6L2 were altered to different degrees in GSE56081 (Figure 7(c)). The results illustrated the value of SMIM1 and SEZ6L2 as important biomarkers of IDD associated with pyroptosis.

### 3.6. The Expression of SMIM1 and SEZ6L2 mRNA

We assessed the mRNA expression of SMIM1 and SEZ6L2 in IDD through an RT-PCR experiment. As shown in Figure 8(a), the expression of SMIM1 mRNA was substantially higher in the severe degenerated NP than in the mild one (*P* < 0.05). As shown in Figure 8(b), the expression of SEZ6L2 mRNA was higher in the SD group than in another (*P* < 0.05). In addition, in the SD group, the expression of IL-1*β* mRNA was significantly increased compared to the MD group (Figure 8(c)). The results of the in vitro experiments are consistent with the above results (Figures 8(d) and 8(e)).

### 3.7. Differential Expression of SMIM1 and SEZ6L2 in Pan-Cancer

We eventually obtained expression data for 34 cancers (Table S3). Among them, SMIM1 indicated a significant upregulation trend in 7 tumors such as BRCA, LUAD, PRAD, SKCM, THCA, OV, and UCS; we observed its significant downregulation in 19 tumors such as GBMLGG, LGG, CESC, STES, KIRP, KIPAN, COAD, COADREAD, STAD KIRC, LUSC, WT, BLCA, TGCT, ALL, LAML, ACC, KICH, and CHOL (Figure 9(a)). SEZ6L2 was observed to be significantly upregulated in 29 tumors such as BRCA, CESC, LUAD, ESCA, STES, KIRP, KIPAN, COAD, COADREAD, PRAD, STAD, HNSC, KIRC, LUSC, LIHC, WT, SKCM, BLCA, THCA, READ, OV PAAD, TGCT, UCS, ALL, LAML, PCPG, ACC, and CHOL; we observed significant downregulation in two tumors such as GBM and KICH (Figure 9(b)). Both SMIM1 and SEZ6L2 are important markers of tumor pan-cancer, with SMIM1 being predominantly downregulated and SEZ6L2 being predominantly upregulated.

### 3.8. Prognostic Value of SMIM1 and SEZ6L2 in Pan-Cancer

SMIM1 was highly expressed in four tumor types (GBMLGG, LGG, CESC, and STAD), and they all showed poor prognosis. In three tumor types (PRAD, MESO, and UVM), SMIM1 was lowly expressed and showed a poor prognosis (Figure 9(c)). The best cutoff value obtained in the survival analysis was 0.3231, based on which the patients were divided into high and low groups, and we finally observed a significant prognostic difference (*P* = 4.3e − 6) (Figure 9(d)). In total, SEZ6L2 displayed a significant prognostic value for 11 tumors. In LAML, CESC, COAD, COADREAD, and GBM5, when SEZ6L2 was highly expressed, it tended to show a poorer prognosis; in GBMLGG, LGG, SKCM, SKCM-M, UVM, and PAAD, its low expression predicted a poorer prognosis (Figure 9(e)). Significant prognostic differences (*P* = 1.8e − 9) were observed in the results of the survival analysis (Figure 9(f)). SMIM1 and SEZ6L2 have an important prognostic value in the pan-cancer analysis.

## 4. Discussion

With changing lifestyles and the growing aging of the population, the prevalence of IDD is increasing year on year and has become a severe threat to the physical and mental health of patients and the economic development of society. Many risk factors for IDD include aging, smoking, obesity, mechanical loading, genetics, hyperglycemia, and hypoxia. Genetic factors have been reported to account for over 70% [21, 22]. IDD is a clinical problem because of the difficulty in early diagnosis and the symptomatic nature of its treatment, which makes it hard to gain a good cure [23, 24]. The helpful news is that with the development of bioinformatics, gene expression profiles can be used to screen for diagnostic biomarkers of disease, providing some clinical convenience and guidance [25–28].

Studies have demonstrated that the intervertebral disc (IVD) is an immune-privileged organ and that immune infiltration plays an important role in developing IDD [29]. In addition, the more severe the IDD, the greater the immune cell infiltration and the more intense the inflammatory response, suggesting that IDD can produce a specific immune microenvironment [30]. Pyroptosis is characterized as inflammatory cellular necrosis, an immune response produced by the body. Various studies have demonstrated the close connection between pyroptosis and immune infiltration [31, 32]. IDD is a complex process in which resident pyroptosis promotes its development [33, 34]. It has been identified that there is a considerable accumulation of inflammatory factors in IDD, leading to the accumulation of NLRP3, caspase-1, GSDMD, and other pyroptosis factors and eventually cell death [35, 36]. Further investigation of the role of pyroptosis-related genes in IDD is consequently required. In this research, SMIM1 and SEZ6L2 were analyzed by bioinformatics and machine learning methods to attain potential biomarkers for IDD diagnosis.

Firstly, we conducted enrichment analysis on DEGs and found that the GO function analysis was mainly enriched in transmembrane receiver protein serine/threonine, kinase signaling pathway, response to lipopolysaccharide, and other biological processes. In contrast, KEGG analysis was mainly enriched in the TGF beta signaling pathway, toll-like receiver signaling pathway, TNF signaling pathway, and other pathways. This is essentially the same as the results of the previous study [37, 38]. The main pathological changes in IDD are apoptosis of the NPCs and degradation of the extracellular matrix [39, 40]. This process has multiple intricate changes, such as inflammatory response, immune response, apoptosis, and autophagy. The DEGs retrieved in this research may also alter IDD through these pathways.

The mechanism of IDD caused by pyroptosis is definite [41]; therefore, this study found that inflammatory factors IL1A, IL1B, NOD2, GBP1, IL6, AK1, EEF2K, and PYCARD were significantly altered in IVD after the intervention. Subsequently, WGCNA analysis was performed to identify the modules associated with cell scorching, and ultimately 11 candidate genes were retrieved from the intersection, namely, SMIM1, FBLN2, ZFP2, B4GALT5, HCRT, SLC6A17, MUSK, SLC26A8, CRHR2, SEZ6L2, and KCNJ15. Machine learning is a powerful tool to perform complex algorithms to detect and diagnose clinical diseases [42, 43]. In this research, the genes were filtered by the LASSO model, and ultimately the value of SMIM1 and SEZ6L2 in the diagnosis of IDD pyroptosis-related genes was clarified by the validation set. Furthermore, we validated RT-PCR on NP tissues with different degrees of degeneration and revealed that SMIM1 and SEZ6L2 mRNA expression was significantly higher in the SD group than in the mild one. The NPCs degeneration model constructed through IL-1*β* also revealed a higher SMIM1 and SEZ6L2 mRNA expression in the degenerated group compared to the control one. This result further illustrates the important value of these two targets in diagnosis and therapy. We subsequently performed a pan-cancer analysis of SMIM1 and SEZ6L2, finding them to be of significant value in cancer diagnosis and prognosis.

The small integral membrane protein 1 (SMIM1) is a limited size red blood cell (RBC) membrane protein whose structure is not thoroughly understood and which is associated with a variety of immune responses [44, 45]. It plays a prominent role in RBC differentiation [46]. Seizure-related 6 homolog like 2 (SEZ6L2) is a type 1 transmembrane protein associated with neurodevelopmental and psychiatric disorders, focusing on neuroimmunological research [47, 48]. It is also an essential regulator mediating lung adenocarcinoma [49] and cholangiocarcinoma [50]. Although no studies have reported these two genes in relation to IDD, a review of the literature indicates that they are both immune-related. Consequently, it is hypothesized that both genes mediate the pyroptosis of NPCs through immune action, which in turn causes IDD. In conclusion, the series of studies presented here demonstrate the important role of SMIM1 and SEZ6L2 in IDD and that they can be used as potential biomarkers for the diagnosis of IDD, which can be further enhanced when combined with imaging and symptomatic examination.

TGF*β* (transforming growth factor-beta) belongs to a group of growth factors that are members of the TGF superfamily and are important in mediating various cellular functions [51]. It has been demonstrated to play a key regulatory role in the molecular biology of IDD [52, 53]. However, the benefits and drawbacks of the TGF-*β* signaling pathway for IDD function remain controversial [54]. Studies have shown that upregulation of TGF*β*1 expression can repair degenerated discs and improve the inflammatory response within the disc, protect against degradation of the extracellular matrix, promote cell proliferation, and reduce cell death [53, 55–58]. Nevertheless, findings in recent years have also shown that over-activation of the TGF-*β* signaling pathway may accelerate the progression of IDD [59–61]. Regardless of the pathogenesis, there is no doubt about the critical role of the TGF*β* signaling pathway in IDD. The enrichment analysis demonstrates the importance of the TFG*β* signaling pathway in IDD, and the bioinformatics results also indicate that both SMIM1 and SEZ6L2 are important diagnostic targets, but the exact relationship between these two has not been reported in the literature. SMIM1 and SEZ6L2 are importantly linked to cellular immunity and inflammation, and the mechanism by which the TGF*β* signaling pathway can regulate IDD by modulating cellular inflammatory responses is also well documented [62, 63]. Therefore, it is hypothesized that the relationship between SMIM1 and SEZ6L2 in the TGF*β* signaling pathway is mainly related to the regulation of cellular inflammatory response and pyroptosis, but the exact mechanism needs to be further explored.

Some limitations exist in this article. Although this study has screened SMIM1 and SEZ6L2 as diagnostic markers for LDD through bioinformatics and machine learning methods, it lacks clinical validation in large samples. Second, it is unclear through which pathway these two genes mediate pyroptosis. In the end, the sample size of the gene set in this research screening the GEO database is small and lacks some conventions, and it needs to be expanded later to improve the quality of the study.

## 5. Conclusion

This research demonstrated the link between IDD and pyroptosis through a bioinformatics approach and combined with machine learning algorithms to identify SMIM1 and SEZ6L2 as important biomarkers, which will help investigate the development pathogenesis of IDD further and identify potential therapeutic targets.

## Figures and Tables

**Figure 1:** Differential mapping analysis of IDD. (a) Chip homogenization histograms; (b and c) PCA plots; (d) volcano plots of DEGs; and (e) thermal plots of DEGs.

**Figure 2:** Bubble diagram for GO and KEGG enrichment analysis of DEGs.

**Figure 3:** A Venn diagram between pyroptosis genes and DEGs. (a) Venn diagram between pyroptosis and Up-DEGs and (b) Venn diagram between pyroptosis genes and Down-DEGs.

**Figure 4:** WGCNA Analysis. (a) Genetic tree diagram; (b) module feature vector clustering heat map; (c, d) analysis of network topologies for various soft threshold powers; (e) and heat map of correlations between module signature genes and differential pyroptosis-related genes.

**Figure 5:** A scatterplot of gene significance (GS) for different pyroptosis genes vs. module membership (MM) in the dark gray and ivory modules.

**Figure 6:** Identification of candidate genes. (a) Venn diagram between WGCNA modules and DEGs; (b) LASSO coefficient profiles of key genes; (c) heat map of correlation analysis between the 11 screened genes; (d) validation of LASSO regression analysis; and (e) ROC curve evaluation of candidate genes.

**Figure 7:** Validation of candidate genes. (a) Heat map of correlation analysis between candidate genes; (b) validation violin map of candidate genes in GSE23130; and (c) validation violin map of candidate genes in GSE56081.

**Figure 8:** The mRNA expressions of candidate genes. (a) The relative mRNA expressions of SMIM1 in NPS; (b) the relative mRNA expressions of SEZ6L2 in NPS; (c) the relative mRNA expressions of IL-1*β* in NPS; (d) the relative mRNA expressions of SMIM1 in NPC; and (e) the relative mRNA expressions of SEZ6L2 in NPC (MD: mild degeneration; SD: severe degeneration; NPS: nucleus pulposus samples; NPC: nucleus pulposus cells) .

**Figure 9:** Pan-cancer analysis of SMIM1 and SEZ6L2. (a) SMIM1 gene expression in pan-cancer; (b) SEZ6L2 gene expression in pan-cancer; (c) prognosis of SMIM1 in pan-cancer; (d) prognosis of SEZ6L2 in pan-cancer; (e) survival curve analysis of SMIM1; and (f) survival curve analysis of SEZ6L2.

**Table 1:** Datasets included for analysis.

Datasets	Platform	Study samples	Control samples
GSE41883	GPL1352	4	4
GSE27494	GPL1352	4	4
GSE23130	GPL1352	8	15
GSE124272	GPL21185	8	8
GSE56081	GPL15314	5	5

## Data Availability

All data are available upon request.

## Supplementary Materials

Supplementary Materials Supplementary Figure S1: differential mapping analysis of IDD. (a) Chip homogenization histograms; (b and c) PCA plots; (d) volcano plots of DEGs; and (e) thermal plots of DEGs (GSE 124272). Supplementary Table S1: SMIM1, SEZ6L2, IL-1*β*, and GAPDH specific primer sequence profile. Supplementary Table S2: 81 pyroptosis-related genes we researched from articles. Supplementary Table S3: abbreviations for cancers' names.
